The article "Effects of transplantation of FGF-2-transfected MSCs and XACB on TNF-α expression with avascular necrosis of the femoral head in rabbits" was published in 2019. Journal: Biosci Rep.

# Effects of transplantation of FGF-2-transfected MSCs and XACB on TNF-α expression with avascular necrosis of the femoral head in rabbits

**DOI:** 10.1042/BSR20180765

**Published:** 2019-04-02

**Authors:** Wuxun Peng, Wentao Dong, Fei Zhang, Jianbo Wang, Jian Zhang, Jianhua Wu, Lei Wang, Chuan Ye, Qing Li, Jin Deng

**Affiliations:** Department of Orthopedics and Trauma, The Affiliated Hospital of Guizhou Medical University, Gui Yang 55000, China

**Keywords:** Avascular necrosis of the femoral head, Bone marrow stromal cells, Basic fibroblast growth factor, Tumor necrosis factor-α, Tissue engineering bone

## Abstract

**Objective:** The present study aimed to investigate the effect of the transplantation of basic fibroblast growth factor (FGF-2) gene-transfected mesenchymal stem cells (MSCs) and xenogeneic antigen-cancellous bone (XACB) on tumor necrosis factor-α (TNF-α) expression with avascular necrosis of the femoral head (ANFH) in rabbits. **Methods:** The models of steroid-induced osteonecrosis in rabbits were randomly divided into five groups: A (model), B (XACB), C (XACB + MSCs), D (XACB + MSCs + LV), and E (XACB + MSCs + LV-FGF-2) groups. The therapeutic effect was evaluated by Hematoxylin and Eosin (H&E) staining. Immunohistochemical and RT-PCR assays were used to detect the protein and mRNA expression of TNF-α in the femoral head, respectively. **Results:** At 12 weeks after the operation, the defect in rabbits in group E was completely repaired, while defects in rabbits in the other groups were not completely repaired, and the area of new bone formation was higher, when compared with the other groups (*P*<0.05). Furthermore, the protein and mRNA expression TNF-α was lower at 3, 6, and 12 weeks after surgery, when compared with the other groups, and the difference was statistically significant (*P*<0.05). **Conclusion:** FGF-2/MSCs/XACB could promote the repair of ANFH, and may be correlated to the inhibition of TNF-α expression.

## Introduction

Avascular necrosis of the femoral head (ANFH) is a hip joint disease characterized by severe shortage of blood supply and intraosseous pressure [1]. In recent years, the incidence of femoral head necrosis has been increasing annually, which has exceeded hip joint tuberculosis and become the first in hip joint diseases [2]. There are many ways to treat femoral head necrosis, such as core decompression, bone grafting, joint formation, and joint replacement [3], and each method has its own shortcomings. Bone marrow stem cells, which are modified or enhanced by gene transfection technology, have become a new and popular treatment plan for the treatment of femoral head necrosis. In the previous experiments conducted by the investigators, basic fibroblast growth factor-2 (FGF-2) gene-transfected mesenchymal stem cells (MSCs) were used to construct tissue-engineered bone to repair the ANFH, which achieved certain results. However, it was found that partial MSC apoptosis occurred after transplantation, and the specific mechanism of apoptosis was not entirely clear. Furthermore, poor nutrition, lack of oxygen, cytokines, and oxidative stress may be involved [4]. In addition, tumor necrosis factor-α (TNF-α), which plays a role in the apoptosis process of MSCs, cannot be ignored. The present study used gene transfection technology to transfect the *FGF-2* gene into rabbit MSCs through the lentiviral vector and cultured this with xenogeneic antigen-cancellous bone (XACB) to produce tissue engineering bone XACB/FGF-2/MSCs, in order to observe the effect of TNF-α on the repair of femoral head defects in rabbits.

## Materials and methods

### Materials

New Zealand white rabbits (Animal Laboratory Center of Guizhou Medical University), DMEM medium (Gibco); FBS (Hyclone), 0.25% pancreatic enzyme plus EDTA (Gilmo); Percoll separation fluid (Sigma), Alkaline phosphatase kit (Beijing Solaibao Technology Co. Ltd.), Antibody CD44 FITC (Beijing Boaosen Biotechnology Co. Ltd.), and a super clean bench (DCM 1 1300, Suzhou); Automatic desktop centrifuge (Ljy25-2, Beijing), CO_2_ incubator (Thermo forma 31I, U.S.A.), Inverted microscope (Olympus), Ndl1000 nucleic acid protein measuring instrument (Nanodrop, U.S.A.), C1000 PCR amplification instrument (Bio-Rad), and an iCycler iQ fluorescence quantitative PCR instrument (Bio-Rad, U.S.A.).

### Methods

#### Separation and culture of rabbit MSCs

Six-week-old male and female New Zealand white rabbits were used, 3% pentobarbital sodium was applied for intravenous anesthesia, and the bone marrow was taken from the femur and tibia of the rabbit using a bone marrow puncture needle. The bone marrow was separated by density gradient centrifugation, and the milky white intercellular layer in the middle was collected. The serum DMEM medium of 10% fetal cow serum containing double resistance was added to be blown into the cell suspension. Then, this was inoculated in a culture bottle, and placed in an incubator at 37°C with 5% CO_2_. After 3 days, the DMEM was changed once after 2–3 days. When cells filled approximately 90% of the bottom of the bottle, the subculture was carried out. Then, the cell morphology was observed using an inverted phase contrast microscope, cellular phenotype CD44 was identified by flow cytometry, and cells were differentiated into osteogenesis *in vitro*.

#### Preparation of tissue engineering of bone

Third-generation rabbit bone marrow stromal stem cells were well grown and used for digestion with pancreatic enzymes. Then, digestion was terminated, cells were centrifuged, the weight of the culture medium was suspended, and the number of cells was counted. According to the MOI value (100) determined by the previous experiment, the virus was added, and the medium was changed after 10 h. The expression of the fluorescent protein was observed using an inverted fluorescence microscope at the later stage, and puromycin was added to obtain the stable strain. The protein expression of FGF-2 was detected by Western blot, and the expression mRNA level of FGF-2 was detected by qPCR. The target cell density was adjusted to ≥ 5 × 10^6^/ml. Pre-treatment was performed in a six-well plate with XACB, and the surface attachment, distribution, and growth of cells were observed using an electron microscope on the sixth day. Then the tissue-engineered bone was obtained.

#### Animal model production and tissue-engineered bone transplantation

According to the methods reported by Wu et al. [5], rabbit models of steroid-induced ANFH were established using endotoxin and methylprednisolone, *Escherichia coli* endotoxin (10 μg/kg) was injected to the ear vein, and repeated after 24 h. Then, the gluteus muscle was injected with methylprednisolone (40 mg/kg) immediately three times, at 24-h intervals. After 6 weeks and MRI screening, the rabbits were randomly divided into five groups. Core decompression and bone tissue implantation were performed according to the group. After anesthetizing with intravenous injection of 3% pentobarbital sodium, the aseptic operation of the lateral incision of the hip was performed. Then, the joint capsule was cut, revealing the femoral head, and holes were drilled at the head and neck junction. The wound was sutured after bone grafting, according to the groupings: group A (model), group B (cancellous bone), group C (XACB + BMSCs), group D (XACB + BMSCs + LV), and group E (XACB + BMSCs + LV-FGF2). Antibiotics were used to prevent infection after surgery. In course of the experiment, the dead animals were filled in the experiment to ensure that 12 samples were available for each group.

#### Histological observation and quantitative analysis of the newborn bone

After post-operative 12 weeks, calcium was taken out of the femoral head using EDTA. Then, conventional dehydration and paraffin embedding were performed, 5-μm thick slices were made, Hematoxylin and Eosin (H&E) staining was performed, and these were observed using a photoscope. A tissue slice was randomly selected for each specimen at each time point to observe the formation of the new bone. Three 100-fold fields of view were randomly selected to observe the new bone formation area. An image observation analysis was performed using the HPIAS-1000 high resolution color pathology image report analysis system to calculate the percentage of the area of new bone formation. The percentage of the area of new bone formation = new bone area/statistical field area (the whole 100-times area) × 100%.

#### Immunohistochemical analysis of TNF-α expression in bone tissue

The immunohistochemical staining of tissue sections in each group at each time point was performed using a TNF-α polyclonal antibody (purchased from Wuhan PhD Bioengineering Co. Ltd.). The number ratio of TNF-α positive cells in each group at each time point was counted using the ImagePro Plus image counting software for statistical analysis.

#### Determination of *TNF-α* mRNA expression levels in femoral head tissue

Real-time fluorescence quantitative-PCR was used for detection. At the 12th week after the operation, four rabbits in each group were killed, and the femoral head tissue was taken. Then, total RNA was extracted by TRIzol, and sized using a reverse transcriptional kit. With TNF-α as the reference gene, the β-actin primer was designed using the Primer Premier software. The β-actin upstream primer was 5′-ATCAGCAAGCAGGAGTAT-3′, while the downstream primer was 5′-CAATCTCGTCTCGTTTCTG-3′. The combined enzyme chain reaction should be 20 μl (2× qPCR Master Mix: 10 μl, upstream and downstream primer: 0.8 μl, cDNA: 2 μl, double steaming water: 6.4 μl). PCR amplification conditions: 95°C modified for 30 s, 95°C degeneration for 10 s, 30 s, and 60°C annealing cycle for 40-times. Each specimen was set-up in two wells for detection, and the numbers were averaged. These data were analyzed using the 2^−ΔΔ*C*^_t_ method.

## Statistical method

SPSS 19.0 statistical software was used for statistical analysis. The normal distribution metering data was indicated by ± S.D., and the comparison between groups was analyzed using single-factor analysis. The LSD test was used for comparison between two groups. *P*<0.05 was considered statistically significant.

## Results

### Culture and identification of MSCs

In our experiments, the MSC characterization and histology staining quality were not satisfactory. We did not put these results in our manuscript. The third-generation BMSCs were spindle-shaped, arranged neatly and fish-like (×100) (Figure 1A). Alizarin Red staining show visible calcium nodules were dyed orange (×100). Alkaline phosphatase staining show the cytoplasm and cytoplasm of dyed positive cells were stained black (×100) (Figure 1B,C). Flow cytometry was used to identify cell surface antigens, and CD44 positive cells were >99% (Figure 1D).

**Figure 1:** Culture and identification of MSCs (**A**) the third-generation BMSCs were spindle-shaped, arranged neatly and fish-like (×100). (**B**) Alizarin Red staining: visible calcium nodules were dyed orange (×100). (**C**) Alkaline phosphatase staining: the cytoplasm and cytoplasm of dyed positive cells were stained black (×100). (**D**) Cell surface antigen CD44 test results: CD44 positive cells were >99%.

### Transfection of BMSCs and detection of *FGF-2* gene transfection

#### Fluorescent protein

A large number of fluorescent green proteins were observed under fluorescence microscopy after the transfection of MSCs (Figure 2A).

**Figure 2:** Transfection of BMSCs and detection of FGF-2 gene transfection (**A**) a large number of fluorescent green proteins were observed under the fluorescence microscopy of transfected BMSCs (×100). (**B**) The mRNA expression level of FGF-2 was detected by qPCR. (**C-D**) The expression level of FGF-2 was detected by Western blot. Compared with the blank group, ^#^*P*<0.05; compared with the Lv-EGFP group, *P<0.05.

#### qPCR test results

The mRNA expression of FGF-2 in transfected BMSCs was higher than that in the empty virus transfection group and blank group (*P*<0.05, Figure 2B).

#### Western blot test results

The protein expression of FGF-2 in transfected BMSCs was higher than that in the empty virus transfection group and blank group (*P*<0.05, Figure 2C,D).

### BMSCs and XACB composite culture

On the sixth day of composite culture, cells were stretched out of pseudopodia under a scanning electron microscope, and extended to the surroundings. The XACB was well grown (Figure 3).

**Figure 3:** BMSCs and XACB composite culture: cells attached to the XACB surface

### MRI screening of the steroid-induced ANFH model

The MRI of the steroid-induced ANFH revealed T1 images with low signal points (Figure 4A) and T2 images with punctuate and patchy high signals (Figure 4B). This was consistent with its MRI diagnosis of positive performance [6].

**Figure 4:** MRI screening of the rabbit model of steroid-induced ANFH (**A**) the model group T1 shows a lower slice of cartilage in the femoral head; (**B**) model group T2 images revealed a patchy high signal at the lower articular cartilage of the femoral head.

### H&E staining and analysis of the area of new bone formation

At 12 weeks after the operation, group A exhibited extensive osteonecrosis, diffused distribution of empty bone lacuna, and fibrous tissue hyperplasia around the necrotic bone (Figure 5A). Group B had a few new bone, and the transplanted bone was not completely absorbed (Figure 5B). In groups C and D, a large number of new bone formations were observed, and the graft bone was absorbed (Figure 5C,D). In group E, a large number of new bone trabeculae were found, which were not clear with normal bone boundaries, and the repair was close to the normal cancellous bone (Fiureg 5E). At 3, 6, and 12 weeks after the operation, the quantitative analysis and comparison of new bone revealed that group E had the largest and significant difference (*P*<0.05, Figure 5F).

**Figure 5:** H&E staining and analysis of the area of the new bone formation (**A**) Group A presented extensive osteonecrosis, diffuse distribution of the empty bone lacuna, and fibrous tissue hyperplasia around the necrotic bone; (**B**) Group B had a few new bone, and the transplanted bone was not absorbed completely; (**C-D**) In groups C and D, a large number of new bone formation was observed, and the graft bone was absorbed; (**E**) In group E, a large number of new bone trabeculae were found, which were not clear with normal bone boundaries, and the repair was close to the normal cancellous bone; (**F**) At 12 weeks after the operation, the quantitative analysis and comparison of new bone revealed that group E had the largest and significant difference. Compared with groups A, B, C and D, ^#^*P*<0.05 (*P*<0.05).

### The mRNA expression level of TNF-α in femoral head tissues

At 12 weeks after the operation, the mRNA expression level of TNF-α in bone tissues in each group revealed the following: this level was significantly higher in group A than in the other groups. When comparison between transplantation groups: group E had the least level, while group B had the greatest level, and the differences were statistically significant (*P*<0.05). There was no significant difference between groups C and D (*P*>0.05, Figure 6).

**Figure 6:** The mRNA expression level of TNF-α in femoral head tissues Compared with groups A, B, C, and D, *P<0.05; compared with group C, ^#^*P*>0.05.

### Immunohistochemical analysis of TNF-α expression

TNF-α antigen-positive cells were dyed brown, the cells were not aligned, and morphological disorders were observed. At 3 weeks, the number ratio of cells with positive expression of TNF-α antigen was the lowest in group E, and the difference was statistically significant (*P*<0.05). At 6 and 12 weeks, the expression of the TNF-α antigen positive cell number ratio in group A was the greatest. The transplantation group: Group E was the least, while group B was the greatest, and the difference was statistically significant, when compared with the other groups (*P*<0.05). There was no significant difference between groups C and D (*P*>0.05, Figure 7).

**Figure 7:** TNF-α immunohistochemistry (**A**–**E**) the staining was strongly positive in groups A–E at TNF-α for 3 weeks, SP ×400. (**F**) At 6 weeks, TNF-α staining in group A was strongly positive, SP ×400. (**G**–**J**) TNF-α staining was moderately positive in groups B–E at 6 weeks, SP ×400. (**K**) At 12 weeks, TNF-α staining in group A was strongly positive, SP ×400. (**L**–**O**) TNF-α staining was weakly positive in groups B–E at 12 weeks, SP ×400. (**P**) At 3, 6, and 12 weeks after the operation, the percentage of TNF-α positive cells in each group is shown. Compared with groups A, B, C, and D, *P<0.05; Compared with group C, ^#^*P*>0.05.

## Discussion

The exact pathogenesis of femoral head necrosis remains unclear. There are a variety of theoretical systems, as well as intravascular coagulation and osteonecrosis theories, fat embolism theories, osteoporosis, and microfractal theories and bone pressure theories [7,8]. The pathological changes are necrosis of bone cells. In the present experiment, glucocorticoid-induced ANFH was used as the model, and its histopathology was characterized by the necrosis of bone marrow cells and the proliferation of adipocytes in the bone marrow, which is consistent with femoral head necrosis pathological changes, and suitable for the treatment of femoral head necrosis. Autologous bone grafting has been regarded as the standard for bone transplantation [9], which was used as the control.

MSCs have been used as seed cells, and the combination of gene transfection and tissue engineering has been the hotspot in the study of femoral head necrosis. MSCs are a kind of pluripotent stem cells in the bone marrow stromal system, which can induce differentiation into bone, cartilage, fat, tendon, nerve, muscle, and other tissues, as well as in the hematopoietic support matrix. It not only carries the target gene, but also plays special cell replacement and cell transformation roles [10–12]. It is an ideal carrier for cell engineering and genetic engineering. In the present experiment, a large number of high-purity MSCs were obtained by density gradient centrifugation combined with the adherent method. The purity of these MSCs was above 95%, and these were successfully differentiated into osteoblasts. FGF-2 has a wide range of biological effects. It not only promotes osteoblasts, chondrocyte protein synthesis, and the cell differentiation and proliferation of other bone growth factor osteogenesis, but also promotes the growth of capillaries, and new bone formation and substitution [13,14]. Studies have shown that transfected bone marrow stromal stem cells do not differ significantly in morphology, and successfully express FGF-2 [15,16]. In the present study, MSCs were transfected by the *FGF-2* gene (MOI = 100), and there was no obvious change in cell morphology, when compared with the control group. Furthermore, the protein expression of FGF-2 increased by approximately 1.8-fold, and the overexpression of this gene was successful. These results were consistent with those reported in the literature.

Scaffolds are mainly used to provide structural support for the cartilage and articular cartilage, in order to prevent collapse in the repair process [17]. The xenogeneic antigen-extracted cancellous bone has good biocompatibility, suitable mechanical strength, natural porous structure, and suitable porosity, which is beneficial to compound seed cells and osteoinductive factors, and facilitates the growth of vascular tissues and osteochondral differentiation [18]. In the present study, the transfected rabbit MSCs were cultured with XACB to obtain tissue engineering bone, and these were used to repair the necrosis of the femoral head. The effect of the transfected BMSCs on the basis of the support of XACB, and from the post-operative 12 weeks of post-operative femoral pathology, was that different degrees of bone formation occurred. However, the tissue-engineered bone formation after transfection was superior to that of the other groups, and the mechanism maybe that the bone marrow stromal stem cells induced the chemotaxis of osteoblasts and osteoclasts after transfection, and promoted the proliferation of osteoblasts [19] and complete bone reconstruction. Inflammation is involved in the repair of ANFH. The study conducted by Samara et al. [20] pointed out that there are a large number of inflammatory factors involved in the development of ANFH, such as IL-1, IL-2, IL-4, IL-6, IL-10, IFN-γ, and TNF-α. TNF-α is an important cytokine for the regulation of bone homeostasis. On the one hand, it causes osteoclastogenesis by activating osteoclasts. On the other hand, it inhibits osteogenic differentiation, and thereby destroys bone tissue [21]. In the experiment, the transplanted group could reduce the number of TNF-α antigen cells in different degrees, and cut down the mRNA expression level of TNF-α. Amongst these groups, group E was superior to the other transplantation groups, and the difference was statistically significant. Furthermore, group E could reduce the number of TNF-α antigen positive cell in the early stage (3 weeks), and the difference was statistically significant. It was speculated that bone marrow stromal stem cells, which were transfected with the FGF-2 gene, could facilitate the growth of capillaries in the early stage and lower the expression of TNF-α, reducing inflammatory response.

In conclusion, tissue-engineered bone with BMSCs as seed cells down-regulated the mRNA level of TNF-α to varying degrees, while tissue-engineered bone XACB/FGF-2/MSCs was superior to other groups. Its mechanism may be the ability to inhibit TNF-α expression, and thereby reducing inflammatory response.

## Abbreviations

ANFH: avascular necrosis of the femoral head
FGF-2: fibroblast growth factor
H&E: Hematoxylin and Eosin
MSC: mesenchymal stem cell
TNF-α: tumor necrosis factor-α
XACB: xenogeneic antigen-cancellous bone
